# MicroRNA Roles in the NF-**κ**B Signaling Pathway during Viral Infections

**DOI:** 10.1155/2014/436097

**Published:** 2014-04-02

**Authors:** Zeqian Gao, Yongxi Dou, Yixia Chen, Yadong Zheng

**Affiliations:** ^1^State Key Laboratory of Veterinary Etiological Biology, Key Laboratory of Veterinary Parasitology of Gansu Province, Lanzhou Veterinary Research Institute, CAAS, Lanzhou, Gansu 730046, China; ^2^College of Life Science and Engineering, Northwest University for Nationalities, Lanzhou 730030, China

## Abstract

NF-**κ**B signaling network is a crucial component of innate immunity. miRNAs are a subtype of small noncoding RNAs, involved in regulation of gene expression at the posttranscriptional level. Increasing evidence has emerged that miRNAs play an important role in regulation of NF-**κ**B signaling pathway during viral infections. Both host and viral miRNAs are attributed to modulation of NF-**κ**B activity, thus affecting viral infection and clearance. Understandings of the mechanisms of these miRNAs will open a direction for development of novel antivirus drugs.

## 1. Introduction

Innate immune system constitutes a first line of defense against inherent and environmental threats and therefore plays a vital role in the early recognition of invading organisms. The NF-*κ*B signaling network, an ancient signaling pathway initially found in unicellular organisms, is a central regulator in innate immunity. Activation of NF-*κ*B signaling cascade relies on germ line-encoded pattern recognition receptors (PRRs) to recognize pathogen derived substances-pathogen associated molecular patterns (PAMPs) [1]. The recognition subsequently triggers a series of proinflammatory responses that alter inflammatory cytokines profiles, thus regulating the host-virus interactions [2].

microRNAs (miRNAs) represent a subclass of small noncoding, regulatory, and single-stranded RNAs and mainly bind to the 3′untranslated region of mRNAs to posttranscriptionally regulate gene expression. miRNAs were first discovered in* Caenorhabditis elegans* [3, 4] and then found to be present in many viruses, animals, and plants, such as Epstein-Barr virus, humans, and Arabidopsis [5–7]. However, the miRNA-mediated silencing pathway may be absent in yeast and some unicellular organisms [8, 9]. miRNAs are mediators of gene silencing via small RNA induced silencing complex (RISC) to induce translational repression or degradation of targeted mRNAs. miRNAs-mediated silencing machinery executes important regulatory functions in multiple cellular processes, including immune responses, cellular proliferation, differentiation, apoptosis, and oncogenic transformation [10–12]. Increasing evidences support the notion that miRNAs also play important roles in modulating NF-*κ*B signaling pathway during viral infections [13–15].

## 2. Biogenesis of Animal miRNAs

In the canonical pathway, the transcription of miRNA genes is performed mostly by RNA polymerase II (Pol II) with a minor proportion of miRNAs that are associated with Alu repeats by RNA polymerase III (Pol III) (Figure 1) [16, 17]. The long primary transcripts (pri-miRNAs) process a 5′cap and 3′polyA tail and form the stem-loop structure which contains a mature miRNA as a part of the double stranded stem connected by a terminal loop [18]. Then, pri-miRNAs are recognized and spliced by Drosha and its cofactor, DiGeorge syndrome critical region gene 8 (DGCR8) in human or Pasha in* Drosophila* and* C. elegans* [16, 19–21]. The cleavage generates a hairpin-structured precursor of miRNAs (pre-miRNAs) with a size of approximately 70 nucleotides. With the help of a nuclear transport receptor (exportin-5) and Ran-GTP, pre-miRNAs are transported from nucleus to cytoplasm [22, 23]. In the cytoplasm, pre-miRNAs are recognized by Dicer, which works in cooperation with human immunodeficiency virus (HIV-1) transactivating response (TAR) RNA binding protein (TRBP or Loquacious in* Drosophila*) to cleave pre-miRNAs into miRNA duplexes [24–28]. Together with Argonaute and other proteins, a miRNA duplex is then loaded to generate RISC [29–31]. The mature miRNA retains, whereas the accompany passenger stand, named miRNA*, is degraded in most cases. Recently, studies have revealed that miRNAs* are also present at a relative level and have the ability to silence targets [32]. Once loaded into the miRNAs-containing RISC, miRNAs serve as a guide to target mRNAs through imperfect sequences complementarities with sites located in the 5′UTR [33, 34], coding regions [35, 36], or 3′-UTR [37], leading to mRNA cleavage or translational repression [38].

In addition to canonical miRNAs, approximately 40% of animal miRNAs, termed as mirtrons, are derived from introns of protein-coding genes [18, 39]. Compared to the canonical pathway, the mirtron production is Drosha-independent to generate pre-miRNAs. The short intron-derived pri-miRNAs are spliced by Spliceosome [40]. The initial splicing products are not linear but are instead of a lariat in which the 3′branchpoint is ligated to the 5′terminus of the intron. With the help of a debranching enzyme, the intron lariats are folded directly to form pre-miRNAs [41, 42]. Afterwards, the intron-derived pre-miRNAs are processed as mentioned in the canonical biogenesis.

Furthermore, there are also several alternative miRNAs biogenesis pathways, such as tRNA-derived miRNAs in mammals, snoRNA-derived miRNAs in* Giardia lamblia*, and AGO-dependent pathway in zebrafish and mammals [43–45].

## 3. Conventional NF-**κ**B Signaling Pathway

NF-*κ*B is a dimeric transcriptional factor, which plays a crucial role in the immediate early pathogen responses and regulates varieties of cellular processes such as inflammation, cellular proliferation, and differentiation [46–48]. NF-*κ*B contains five members NF-*κ*B1 or p50, NF-*κ*B2 or p52, c-Rel, RelA or p65, and RelB, all of which belong to Rel family. These five members can be classified into two groups: one consists of c-Rel, p65, and RelB, which are synthesized as an active form, and the other includes p50 and p52, which are proteolytically processed from precursor subunits, p100 and p105, respectively [49]. The five Rel proteins share a Rel homology domain (RHD), which is essential for binding to cognate DNA elements and nuclear translocation as well as dimerization to the other members of NF-*κ*B proteins [50]. All NF-*κ*B proteins can form homodimers or heterodimers with an exception of RelB that can only form heterodimers [51]. In most quiescent cells, a p50–p65 heterodimer is the predominant form and bound to I*κ*B*α*, of which the ankyrin repeats interact with the DNA-binding region. Moreover, binding of p50–p65 to I*κ*B*α* also masks the nuclear localization signals (NLSs) of p50–p65 and then sequesters the p50–p65-I*κ*B*α* complex in the cytoplasm, making NF-*κ*B inactive [52].

Activation of NF-*κ*B signaling pathway is initiated in response to extracellular stimuli, including viral and bacterial infection, exposure to proinflammatory cytokines, and stress-inducing agents. These stimuli are recognized by different kinds of pattern recognition receptors (PRRs) and transmitted into the cell. The altered conformation of PRRs caused by extracellular stimuli triggers the recruitment of myeloid differentiation primary response gene 88 (MyD88) [53]. This adaptor protein recruits a variety of downstream components and initiates the signaling cascade. The signaling cascade culminates in the activation of I*κ*B kinases (IKKs). IKKs are a multisubunit complex, consisting of two catalytic subunits (IKK*α* and IKK*β*) and the NF-*κ*B Essential Modulator (NEMO or also termed IKK*γ*) noncatalytic accessory subunit [54]. The NF-*κ*B-I*κ*B complex is activated by IKKs through the phosphorylation of I*κ*B [55]. This phosphorylation facilitates ubiquitin-dependent degradation of I*κ*B by 26S proteasome, releasing NF-*κ*B from the inhibitory complex and allowing translocation of NF-*κ*B dimers to the nucleus and activation of target gene transcription [56].

## 4. Regulation of NF-**κ**B Signaling Pathway by miRNAs during Viral Infections

Increasing evidences have emerged that viral infections can alter expression of cellular miRNAs that are involved in regulation of NF-*κ*B [57]. At the same time, viral miRNAs are also active in modulation of immune responses via direct targeting of NF-*κ*B (Figure 2 and Table 1). The interaction between viruses and host cells needs to initially recognize viruses by PRRs. Thus, exact control of PRRs expression by miRNAs is one of the approaches to modulate the NF-*κ*B signaling pathway. After HIV and Kaposi's sarcoma-associated herpesvirus (KSHV) stimulation, all the members of Let-7 family and miR-223 were downregulated. Reduced Let-7 and miR-223 gave rise to an increase of TLR3 and TLR4 expression, resulting in excessive inflammation and tissue damage [58]. Recent studies have revealed that miR-146 is also involved in regulation of TLR4 [59]. miR-146 was first functionally identified as an immune response regulator that had impacts on mammalian responses to microbial infections. miR-146 was found to be involved in regulation of Interleukin-1 receptor-associated kinase 1 (IRAK1) and TNF receptor-associated factor 6 (TRAF6), downstream molecules of MyD88, and to be expressed under the control of NF-*κ*B signaling pathway [60]. These suggest the presence of a negative regulatory network, in which HIV and hepatitis C virus (HCV) infections upregulate miR-146 and miR-21 that in turn downregulate IRAK1 and TRAF6 to reduce the activity of NF-*κ*B [61, 62].

Accumulating evidence has demonstrated that miR-155 can negatively regulate NF-*κ*B signaling pathway by targeting different key signaling protein genes. The adaptor protein MyD88 has been identified as one of the targets, and overexpression of miR-155 results in significantly reduced IL-8 synthesis induced by* Helicobacter pylori* infection [63]. It was also documented that MyD88 was targeted by other miRNAs, including miR-200b/c and miR-21 [61, 64]. In the HCV or HIV infected cells, the expression of miR155 and miR-21 was upregulated, leading to repression of NF-*κ*B signaling pathway [65–67]. However, miR-200b/c were downregulated in the HCV or HIV infected cells [68, 69]. So far, it is not fully clear what makes the difference of those miRNA genes' expressions.

TGF-*β*-activating kinase 1 (TAK1) forms a complex with TAK1-binding protein 1 (TAB1) and TAK1-binding protein 2 (TAB2), which modulates the activity of IKK*β*. Evolutionarily conserved miR-10a binding sites were identified in TAK1. miR-10a is able to target TAK1 transcripts, increasing the total expression of I*κ*B and impairing NF-*κ*B activation [70]. Expression of TAB2, a signal molecule downstream of TRAF6, was also regulated by the same miRNAs as ones involved in regulation of MyD88. For instance, miR-155 is able to bind to the 3′UTR of TAB2 transcripts, resulting in activation of mitogen-activated protein kinases (MAPK) kinases [71]. IKKs, downstream signal molecules of TAK1, are predominantly present in the form of which consists an IKK*α*-IKK*β* heterodimer and NEMO subunit. IKK*α* was recently shown to be targeted by miR-16 and -223 and IKK*β* targeted by miR-199, leading to negative regulation of NF-*κ*B signaling pathway [72, 73].

In addition to the direct targeting of the components of NF-*κ*B signaling pathway, miRNAs can also target regulatory molecules, such as Cylindromatosis (CYLD) [74], mothers against decapentaplegic homolog 7 (SMAD7) [75], and NF-*κ*B repressing factor (NFR) [75, 76], to modulate the NF-*κ*B signaling pathway indirectly. The tumor suppressor, programmed cell death protein 4 (PDCD4), is a proinflammatory protein that promotes activation of NF-*κ*B through an unknown mechanism. miR-21 has been shown to inhibit both NF-*κ*B activities via targeting PDCD4 and expression of other proinflammatory factors [77].

The major consequence of NF-*κ*B activation is the production of inflammatory cytokines, which are crucial in virus clearance and inflammatory cell recruitment to infectious sites. Cytokine genes can be targeted directly by miRNAs (Figure 2). For instance, IL-12p35 can be targeted by miR-21 in macrophages and dendritic cells, resulting in restricted adaptive Th1 responses [78]. In addition to host miRNAs, virus-encoded miRNAs have also found ways to modulate NF-*κ*B signaling cascade (Table 1). For instance, KSHV encodes miRNAs, miR-K1, miR-K5, and miR-K9 that directly target I*κ*B*α*, MyD88, and IRAK1, thus regulating the NF-*κ*B signaling pathway [79, 80].

## 5. Perspectives

During viral infections, miRNAs serve as posttranscriptional regulators of gene expression in virus replication and host's immune responses. A number of miRNAs are known to be involved in regulation of the NF-*κ*B signaling pathway through multiple steps, thus affecting viral infection outcomes. Some miRNAs have been shown to play bilateral roles in viral clearance and replication. For instance, during HIV infection downregulation of miR-16 results in the promotion of NF-*κ*B signaling pathway, thus enhancing the level of immune responses [73]. However, downregulation of miR-16 also increases the HIV-1 replication via indirectly promoting the translation of its target gene, Pur-*α* [81]. The precise mechanisms whereby the host regulates the expression of miR-16 to balance the viral clearance and replication are not fully understood. Further studies will be required to investigate the regulatory network for regulation of miR-16, which increases our understanding of molecular mechanisms of viral infections.

## Figures and Tables

**Figure 1:** Biogenesis of canonical and mirtron miRNAs in animal cells. In canonical pathway, miRNA genes are transcribed by RNA polymerase Π (Pol Π) or RNA polymerase *Ш* (Pol *Ш*) to produce the primary miRNA (pri-miRNA) transcripts. The cropping of pri-miRNAs is mediated by the Drosha-DGCR8 complex (viz. microprocessor) that generates 60–70 nt precursor miRNAs (pre-miRNAs). After being exported by exportin-5 from the nucleus, pre-miRNAs are processed into ~22 nt miRNA/miRNA* duplexes by Dicer-TRBP complex. Finally, mature miRNAs are loaded onto Argonaute proteins, leading to cleavage or degradation of the targeted genes. In the mirtron pathway, the miRNA-containing introns, termed as mirtrons, are spliced and debranched into pre-miRNAs that bypass Drosha processing. Afterwards, the intron-derived pre-miRNAs access the canonical miRNA pathway during nuclear export and then are spliced by Dicer and loaded onto Argonaute proteins.

**Figure 2:** Canonical NF-*κ*B signaling network regulated by miRNAs. PRRs are activated by different types of pathogens and initiate signaling transduction to induce the production of inflammatory cytokines. Host- or virus-derived miRNAs are involved in delicate regulation of the pathway at multiple levels. PRRs: pattern recognition receptors; MyD88: myeloid differentiation primary response gene 88; IRAK: Interleukin-1 receptor-associated kinase; TRAF: TNF receptor-associated factor; CYLD: Cylindromatosis; TAB: TAK1-binding protein; TAK: TGF-*β*-activating kinase; NEMO: NF-*κ*B Essential Modulator or IKK*γ*; PENT: phosphatase and tensin homologue; SMAD7: mothers against decapentaplegic homolog 7; PDCD4: programmed cell death protein 4; NFR: NF-*κ*B repressing factor.

**Table 1:** miRNAs involved in viral infections via regulation of NF-*κ*B.

miRNA genes	Origin	Expression	Targets	Reference
miR-21	Host	Up	MyD88, IRAK1, PTEN, SMAD7, PDCD4, and IL-12p35	[61, 66, 77, 78, 82–84]
miR-155	Host	Up	MyD88, TAB2, and IKK*ε*	[63, 85, 86]
miR-199a	Host	ND	IKK*β*	[87, 88]
miR-146	Host	Up	IRAK1, IRAK2, and TRAF6	[60, 83, 84, 89]
miR-200b/c	Host	Down	MyD88	[64]
miR-301a	Host	Down	NKFR	[90, 91]
miR-181	Host	Up	CYLD	[74, 92]
miR-16	Host	Down	IKK*α* and TNF-*α*	[73, 93]
miR-223	Host	Down	TLR3, TLR4, STAT3, and IKK*α*	[73, 94–97]
miR-125b	Host	Down	TNF-*α*	[85, 98]
miR-210	Host	Up	NF-*κ*B1	[70, 99]
miR-10a	Host	Up	TAK1	[70, 99]
Let-7	Host	Down	IL-6 and TLR-4	[100, 101]
miR-K5	Virus	Up	MyD88	[79]
miR-K9	Virus	Up	IRAK1	[79]
miR-K12-1	Virus	Up	I*κ*B*α*	[80]

Note: “Up”: upregulated; “Down”: downregulated; “ND”: not determined.
